# Efficacy of Low Molecular Weight Heparin in Preventing Perinatal Venous Thrombosis: A Meta-Analysis

**DOI:** 10.1155/2022/1248577

**Published:** 2022-07-26

**Authors:** Yan Huang, Fei Li, Changhong Li, Xueli Liao

**Affiliations:** ^1^Department of Obstetrics, Hainan Women and Children's Medical Center, Haikou 570216, China; ^2^Department of Obstetrics and Gynecology, Chengmai County People's Hospital, Chengmai 571900, China; ^3^Department of Pharmacy, Hainan Women and Children's Medical Center, Haikou 570216, China

## Abstract

**Background:**

There have been controversies about the preventive effect of low molecular weight heparin (LMWH) on venous thrombosis (VT) in the perinatal period. This study is aimed at exploring the effectiveness of LMWH in preventing perinatal VT through meta-analysis.

**Methods:**

Databases such as CNKI, China Biology Medicine disc (CBMdisc), Wanfang, PubMed, MEDLINE, Embase, and Central were searched. Inclusion criteria were as follows: (1) subjects: women at high risk of perinatal VT; (2) experimental group and control group; (3) intervention measures: the experimental group was given LMWH, while the control group was given placebo or standard heparin or physical therapy; (4) outcomes: perinatal VT events or bleeding events; and (5) randomized controlled trials (RCTs). Jadad scale was used to evaluate the literature quality. The Mantel-Haenszel method was used to calculate the odds ratio (OR) and 95% confidence interval (CI). The chi-square test was used to analyze the heterogeneity of the included literature. Subgroup analysis was used to explore the source of heterogeneity. Publication bias was evaluated via funnel plot and Egger test.

**Results:**

The incidence of perinatal VT in the LMWH group was lower than that in the control group (OR = 0.16, 95% CI (0.08, 0.32), *P* < 0.00001). There was no heterogeneity among literatures (*P* = 0.77, *I*^2^ = 0%) and no publication bias. The incidence of postpartum VT in the LMWH group was lower than that in the control group (OR = 0.14, 95% CI (0.07, 0.30), *P* < 0.00001). There was no heterogeneity among literatures (*P* = 0.69, *I*^2^ = 0%) and no publication bias. The incidence of perinatal bleeding in the LMWH group was higher than in the control group (OR = 1.72, 95% CI (1.06, 2.77), *P* = 0.03). There was no heterogeneity among literatures (*P* = 0.25, *I*^2^ = 26%) and no publication bias.

**Conclusion:**

LMWH can reduce the incidence of perinatal VT in high-risk women but increase the risk of bleeding. The use of LMWH to prevent perinatal VT should be closely monitored.

## 1. Introduction

Perinatal venous thromboembolism (VT) is the leading cause of maternal death in developed countries [1–3]. The increase in gestational weeks increases the risk of VT [4, 5], and the peak period of VT occurs within 6 weeks after delivery [6]. However, the pathogenesis of VT is not clear. VT is a disease caused by multiple factors [7–9], which may be related to specific gene expression [10, 11]. In addition, pregnancy itself is a high-risk factor for VT [3–5, 12]. Changes in estrogen and progesterone levels during pregnancy lead to vasodilatation of lower limb veins [3, 5]. The enlarged uterus oppresses the pelvic vein and causes blood stasis [4, 5]. Coagulation factors are activated during pregnancy, and the serum level is significantly increased [5]. A series of physiological changes significantly increased the risk of perinatal VT. Besides, the perinatal period is often associated with many other clinical risk factors, such as obesity, braking, history of VT, and cesarean section. When multiple risk factors are superimposed, pregnant women need closer monitoring and timely preventive measures [3].

The anticoagulation effect of low molecular weight heparin (LMWH) is better than that of unfractionated heparin by reducing the risk of bleeding [13–15]. Compared with unfractionated heparin, complications such as osteoporosis and thrombocytopenia are rarer in patients using LMWH [15, 16]. Therefore, LMWH is easy to use, with high bioavailability, a long half-life, stable pharmacokinetics, and no need for frequent monitoring [17, 18].

Previous studies have been controversial about the preventive effect of LMWH on perinatal VT. Studies [19] have pointed out that LMWH cannot reduce the incidence of perinatal VT events and may increase the risk of bleeding. Other studies [20] held different views. LMWH could effectively prevent VT events in high-risk pregnant women after cesarean section and reduce fibrinogen levels [20]. Therefore, we conducted a meta-analysis to explore the preventive effect of LMWH on perinatal VT.

## 2. Materials and Methods

### 2.1. Literature Search

We searched in CNKI, China Biology Medicine disc (CBMdisc), Wanfang, PubMed, Medline, Embase, Central, and other databases. The search terms included low molecular weight heparin, enoxaparin, nadroparin, dalteparin, tinzaparin, pregnancy, perinatal stage, postpartum, venous thrombosis, thrombogenesis, and thromboembolism. The deadline for the literature search was June 1, 2022. No document language was limited.

### 2.2. Literature Screening

Inclusion criteria were as follows: (1) subjects: perinatal VT high-risk women. Pregnant women with one or more of the following risk factors are considered to be a population with high risk of perinatal VT: history of thromboembolism, gestational hypertension, diabetes, advanced age, obesity, multiple births, or smoking; (2) the experimental group and the control group were set up; (3) intervention measures: the experimental group was given LMWH to prevent perinatal VT, and the control group was given placebo or unfractionated heparin or physical therapy to prevent perinatal VT; (4) outcomes: including perinatal VT events or bleeding events; and (5) randomized controlled trials (RCTs).

Exclusion criteria were as follows: (1) repeated reports, (2) animal experiments, (3) the subjects received other anticoagulant drugs, (4) observational studies, and (5) the key data in the literature were missing and could not be supplemented.

### 2.3. Data Extraction and Literature Quality Evaluation

Researchers read the full text and extracted the data. The extracted contents included the number of cases, basic diseases, mode of delivery, intervention measures, drug types, drug doses, the incidence of VT, and bleeding events. The Jadad scale was used to evaluate the quality of literature, including the generation of random groups, randomized hidden blind method, implementation of a blind method, loss of follow-up, and withdrawal. Two researchers carried out the above work independently and made crosscomparison after completing the work. If there were differences, the two authors discussed and reached an agreement.

### 2.4. Statistical Analysis

The results of the included studies were meta-analyzed using the Cochrane software RevMan5.3. Odds ratio (OR) and 95% confidence interval (CI) were used as effect quantities. OR and 95% CI were calculated using the Mantel-Haenszel statistical method. The chi-square test was used to analyze the heterogeneity of the included literature. *I*^2^ < 50% and *P* > 0.10 indicated no heterogeneity among the literature, and the fixed effect model was used. *I*^2^ ≥ 50% or *P* ≤ 0.10 indicated heterogeneity among the literature. Subgroup analysis was used to explore the source of heterogeneity. If it was impossible to clarify the heterogeneity source and eliminate it, the literature results were combined or summarized using the random effect model. A funnel test was used to evaluate publication bias. Two-way *P* < 0.05 meant statistically significant.

## 3. Results

### 3.1. Literature Screening

A total of 674 literatures were retrieved. According to the inclusion and exclusion criteria, 663 literature were excluded, and 11 literature were included in this meta-analysis [19–29]. This study included 1512 high-risk women with perinatal VT, with 758 cases in the LMWH group and 754 cases in the control group. The flow chart of literature screening is shown in Figure 1. The literature characteristics and quality evaluation are shown in Table 1.

### 3.2. LMWH and the Incidence of Perinatal VT

10 studies involved the efficacy of LMWH in preventing perinatal VT. There was no heterogeneity among the literature (chi^2^ = 4.93, *P* = 0.77, *I*^2^ = 0%), and the fixed-effect model was used. The incidence of perinatal VT in the LMWH group was lower than that in the control group (OR = 0.16, 95% CI (0.08, 0.32), *Z* = 5.19, *P* < 0.00001), as shown in Figure 2. The funnel chart showed that the scatter points were distributed within the confidence interval, which was roughly symmetrical, and there was no publication bias, as shown in Figure 3.

### 3.3. LMWH and the Incidence of Postpartum VT

A total of 7 studies involved the efficacy of LMWH in preventing postpartum VT. There was no heterogeneity among the literature (chi^2^ = 3.92, *P* = 0.69, *I*^2^ = 0%), and the fixed-effect model was used. The incidence of postpartum VT in the LMWH group was lower than that in the control group (OR = 0.14, 95% CI (0.07, 0.30), *Z* = 5.11, *P* < 0.00001), as shown in Figure 4. The funnel chart shows that the scatter points were distributed within the confidence interval, which was roughly symmetrical, and there was no publication bias, as shown in Figure 5.

### 3.4. LMWH and the Incidence of Perinatal Hemorrhage

A total of 5 studies involved the effect of LMWH on the incidence of perinatal hemorrhage. There was no heterogeneity among the literature (chi^2^ = 5.40, *P* = 0.25, *I*^2^ = 26%), and the fixed-effect model was used. The incidence of perinatal hemorrhage in the LMWH group was higher than that in the control group (OR = 1.72, 95% CI (1.06, 2.77), *Z* = 2.21, *P* = 0.03), as shown in Figure 6. The funnel chart showed that the scatter points were distributed within the confidence interval, which was roughly symmetrical, and there was no publication bias, as shown in Figure 7.

## 4. Discussion

Rodger et al. [19] showed that the use of LMWH failed to reduce the incidence of venous thrombosis and abortion. There was no difference in the incidence of major bleeding events between the LMWH group and the control group, but minor bleeding events were more common in the LMWH group. Badawy et al. [21] have shown that LMWH can reduce the incidence of early abortion and late abortion. There was no significant difference between the LMWH group and control group in pregnancy mode, amount of bleeding during production, and incidence of placental abruption. Their study also pointed out that the average weight of newborns in the LMWH group was higher than that in the control group. They showed that continuous use of LMWH during pregnancy is safe and can reduce the incidence of spontaneous abortion. Burrows et al. [23] conducted a multicenter prospective trial in a pilot study. In this study, patients in the control group were more likely to receive general anesthesia. In addition, the baseline data were balanced. Their results showed that the efficacy of LMWH and the control group in preventing the incidence of VT after a cesarean section was similar. They also pointed out that multicenter RCTs were feasible. Gates et al. [24] showed no difference in the incidence of thromboembolic events and bleeding events between the two groups. Pettilä et al. [28] showed no VT event in the control and LMWH groups. There was no significant difference between the two groups in the incidence of other complications, including osteoporotic fractures, massive bleeding, blood transfusion, spontaneous abortion, and cesarean section. The incidence of minor bleeding events in the LMWH group was lower than in the control group. Pettilä et al. displayed that LMWH has good safety and can be used for VT event prevention. Zhang [29] showed that the possibility of bleeding caused by low molecular weight heparins is lower than that of unfractionated heparin, and the anticoagulation effect is better. LMWH is easy to use, with high bioavailability and fewer adverse reactions. Their results showed that routine subcutaneous injection of low molecular weight heparin sodium after cesarean section in high-risk pregnant women with VT could effectively prevent the occurrence of venous thrombosis in lower limbs. Huang [20] considered that the incidence of deep venous thrombosis of lower limbs in the LMWH group was 3.23%, and that in the control group was 22.58%. There was a significant difference between the two groups. There was no significant difference in platelet count, prothrombin time, and activated partial thrombin time between the LMWH group and control group. The fibrinogen level in the LMWH group was lower than that in the control group. LMWH could effectively prevent VT events in high-risk pregnant women after cesarean section and shorten the rehabilitation time. Bi [22] showed that the incidence of lower limb VT was 17.18% in the control group and 2.22% in the LMWH group. LMWH has a very superior preventive effect on lower extremity deep venous thrombosis in high-risk pregnant women after cesarean section. Liu [27] conducted RCTs to explore the preventive effect of LMWH combined with physical therapy on thrombotic diseases in high-risk pregnant women after cesarean section. The incidence of lower limb VT in the experimental group was lower than that in the control group. The fibrinogen level in the experimental group was lower than that in the control group. Li et al. [25] showed no VT event in the LMWH group. In comparison, 11 patients (21.57%) had deep venous thrombosis in the control group. Therefore, LMWH reduces VT risk. 6 days after cesarean section, the levels of D-dimer and fibrinogen in the LMWH group were significantly lower than those in the control group. They indicated that LMWH has the advantages of no drug monitoring, a long half-life, and no adverse reactions such as bleeding, easy absorption, and moderate price and can effectively prevent the occurrence of deep venous thrombosis after cesarean section. Lin et al. [26] showed that LMWH can improve blood coagulation and hemorheology of high-risk pregnant women after cesarean section, reduce lower limb pain and swelling, restore skin color, and reduce the incidence of lower limb deep venous thrombosis without noticeable adverse reactions.

As can be seen from the above review, the results of our included studies are not completely consistent. In our analysis, there may be some reasons as follows. Firstly, the sample size of the single study is small, which may lead to sample selection bias. Secondly, differences in dose and regimen may influence the results. Finally, the level of local care may influence the perinatal complication rate. We resolved these controversies through meta-analysis. Our meta-analysis showed that LMWH could reduce the incidence of perinatal and postpartum VT and increase the incidence of perinatal hemorrhage in women at high risk of VT.

In addition to preventing VT, some meta-analyses confirmed the efficacy of LMWH in other perinatal diseases. Jiang et al. [30] figured out that LMWH can effectively treat unexplained recurrent abortion. Sirico et al. [31] showed that LMWH does not increase the risk of bleeding and the incidence of blood transfusion during pregnancy. The result was not consistent with ours. This study did not select pregnant women at high risk of VT, but all pregnant women, as subject. Cohort study, case control study, and randomized controlled study were included in this study. This may result in low credibility of the conclusions. Roberge et al. [32] displayed that the combination of LMWH and aspirin can significantly reduce the incidence of preeclampsia and preterm birth.

In conclusion, LMWH can reduce the incidence of perinatal VT in women with high-risk VT but increase the risk of bleeding. When using LMWH to prevent perinatal VT, maternal should be closely monitored.

## Figures and Tables

**Figure 1:** Document screening flow chart.

**Figure 2:** Forest map: comparison of perinatal VT incidence between the LMWH group and control group. LMWH: low molecular weight; VT: venous thrombus embolism.

**Figure 3:** Funnel chart: comparison of perinatal VT incidence between the LMWH group and control group. OR: odds ratio.

**Figure 4:** Forest map: comparison of the incidence of postpartum VT between the LMWH group and control group. LMWH: low molecular weight; VT: venous thrombus embolism.

**Figure 5:** Funnel chart: comparison of the incidence of postpartum VT between the LMWH group and control group. OR: odds ratio.

**Figure 6:** Forest map: comparison of perinatal bleeding rate between the LMWH group and control group. LMWH: low molecular weight; VT: venous thrombus embolism.

**Figure 7:** Funnel chart: comparison of perinatal bleeding rate between the LMWH group and control group. OR: odds ratio.

**Table 1:** Basic characteristics and Jadad score of included literature.

Author	Year	No. of patients		Study type	Intervention		Outcomes	Jadad
		LMWH	Control		LMWH	Control		
Badawy et al. [21]	2008	170	170	RCT	Enoxaparin sodium (0.2 ml, once daily) + folic acid tablets (0.5 mg daily)	Folic acid tablets (0.5 mg daily)	Hemorrhage	6
Bi [22]	2017	45	45	RCT	LMWH sodium (twice daily) + PT	PT	Postpartum VT	4
Burrows et al. [23]	2001	39	37	RCT	Dalteparin (2,500 IU, once daily)	Normal sodium	Postpartum VT; hemorrhage	6
Gates et al. [24]	2004	78	79	RCT	Enoxaparin (40 mg, once daily)	Placebo (1 ml, once daily)	Perinatal VT; hemorrhage	7
Huang [20]	2018	31	31	RCT	LMWH sodium (200 U/kg, once daily) + PT	PT	Perinatal VT	4
Li et al. [25]	2018	51	51	RCT	Enoxaparin (40 mg, once daily) + obstetrical care	Obstetrical care	Postpartum VT	3
Lin et al. [26]	2021	58	58	RCT	LMWH sodium (5000 U/kg, once daily)	Conventional therapy	Postpartum VT	4
Liu [27]	2020	32	32	RCT	LMWH sodium (4250 U/kg, twice daily) + PT	PT	Postpartum VT	3
Pettilä et al. [28]	1999	50	50	RCT	Dalteparin once daily (mean 4631 IU/day)	Unfractionated heparin twice daily (20569 IU/day)	Perinatal VT; hemorrhage	5
Rodger et al. [19]	2014	146	143	RCT	Dalteparin: 5000 IU once daily + obstetrical care	Obstetrical care	Perinatal VT; hemorrhage	6
Zhang [29]	2013	58	58	RCT	LMWH sodium (5000 U/kg, twice daily)	Conventional therapy	Postpartum VT	4

Note: LMWH: low molecular weight heparin; RCT: randomized controlled trial; PT: physical therapy; VT: venous thrombosis.

## Data Availability

The data used to support the findings of this study are available from the corresponding author upon request.
